The article "Tibetan Medicine Shi-Wei-Gan-Ning-San Alleviates Carbon Tetrachloride-Induced Chronic Liver Injury by Inhibiting TGF-β1 in Wistar Rats" was published in 2022. Journal: Evid Based Complement Alternat Med.

# Tibetan Medicine Shi-Wei-Gan-Ning-San Alleviates Carbon Tetrachloride-Induced Chronic Liver Injury by Inhibiting TGF-*β*1 in Wistar Rats

**DOI:** 10.1155/2022/2011876

**Published:** 2022-08-16

**Authors:** Ziming Jia, Yanhua Zheng, Shaohua Fu, Jingjing Qu, Jie Tian, Wen Qu, Zhinan Mei

**Affiliations:** ^1^Hubei Provincial Key Laboratory for Applied Toxicology, Hubei Provincial Center for Disease Control and Prevention, Wuhan 430079, China; ^2^College of Pharmaceutical Sciences, South-Central University for Nationalities, Wuhan 430074, China

## Abstract

**Background:**

Shi-Wei-Gan-Ning-San (SWGNS) is a classic Tibetan prescription, which has obvious clinical effects in the treatment of viral hepatitis, fatty liver, liver fibrosis, liver cirrhosis, liver cancer, and other liver injuries. However, animal studies and mechanism studies are still lacking. This study aimed to investigate its hepatoprotective efficacy and pharmacological mechanism in animal experiments.

**Methods:**

Chronic liver injury was induced by oral administration of carbon tetrachloride (CCl_4_) in Wistar rats for 13 weeks. SWGNS was administered orally to rats at doses of 235, 705, and 1410 mg/kg for 13 weeks. Blood samples were collected for biochemical, ELISA, and radioimmunoassay. Livers were harvested for H&E and immunohistochemical staining. The major constituents of SWGNS were analyzed by HPLC. In vitro experiments were used to explore the protective effect of Crocin on BRL-3A in the environment of H_2_O_2_.

**Results:**

SWGNS reversed weight loss is induced by CCl_4_. Serum assays showed that SWGNS reduced CCl_4_-induced alanine aminotransferase, aspartate aminotransferase, total bilirubin, and *γ*-glutamyltransferase levels and increased the total protein and albumin levels. Histopathological evaluation showed that SWGNS alleviated hepatic steatosis, fibrosis, and inflammation. Furthermore, SWNGS reduced CCl_4_-induced elevations of TGF-*β*1, hyaluronic acid, laminin, and collagen IV in serum and reduced the high expression of *α*-SMA in tissues. Moreover, Crocin I and II are the main components of SWGNS. Crocin attenuated the damaging effects of H_2_O_2_ on BRL-3A.

**Conclusions:**

In conclusion, SWGNS alleviated CCl_4_-induced chronic liver injury by inhibiting the TGF-*β*1 pathway. This plays an important role in promoting traditional Tibetan medicine in clinical practice.

## 1. Introduction

The liver is an important metabolic organ in the body. It performs an important role in the metabolism, transformation, and detoxification of various endogenous and exogenous substances. Liver injury and liver diseases are one of the most dangerous diseases that are a threat to human life [1–3]. Traditional Chinese medicine (TCM) has shown a good hepatoprotective effect on various chronic liver diseases clinically [4]. Although, TCM has been used in Eastern medicine for thousands of years; however, there is a lack of scientific evidence data on its therapeutic benefits.

The article "Tibetan Medicine Shi-Wei-Gan-Ning-San Alleviates Carbon Tetrachloride-Induced Chronic Liver Injury by Inhibiting TGF-β1 in Wistar Rats" was published in 2022. Journal: Evid Based Complement Alternat Med.

Liver injury can be classified as acute or chronic and is caused by a variety of different pathogens, such as chemicals, drugs, viruses, and toxins. Liver fibrosis, the final common stage of most chronic liver diseases, was once considered incurable. However, this view is changing in recent years, and some early-stage liver fibrosis can be reversed. Liver fibrosis is closely related to chronic liver injury and subsequent inflammatory response [5]. Inflammatory cytokines in the liver drive the activation of hepatic stellate cells (HSCs), the primary cells responsible for liver fibrosis. Transforming growth factor-*β*1 (TGF-*β*1) is an important profibrotic mediator that activates HSCs to upregulate the expression of hyaluronic acid (HA), laminin (LN), collagen IV (CIV), and *α*-smooth muscle actin (*α*-SMA) [6, 7]. In addition, the expression level of extracellular matrix (ECM) has also been considered a specific biomarker of liver fibrosis. Therefore, these factors are considered sensitive indicators of liver injury.

Traditional Tibetan medicine is one of the oldest well-known medical systems with a long history of more than 2000 years [8]. Shi-Wei-Gan-Ning-San (SWGNS) is a traditional Tibetan medicine formulation that has been used for the treatment of liver fibrosis for many years and has shown hepatoprotective effects in clinical applications [9–11]. The formula consists of seven herbs (*Carthamus tinctorius*, *Crocus sativus*, *Herpetospermum pedunculosum*, *Meconopsis integrifolia*, *Dracocephalum tanguticum*, *Saxifraga stolonifera*, and *Corydalis impatiens*) and five mineral medicines (bear gallbladder, Calculus Bovis, Brag-zhun, Calciosinti, and Turquoisis). Although it has been used clinically for many years as an empirical formulation, however, little experimental data are available on its efficacy and underlying mechanisms. The lack of scientific data for SWGNS limits its broad clinical application.

This study aimed to investigate the efficacy of SWGNS on carbon tetrachloride (CCl_4_)-induced chronic liver injury in Wistar rats and to explore the underlying mechanisms. We hypothesized that SWGNS alleviated CCl_4_-induced chronic liver injury by reducing TGF-*β*1 expression. To this end, we collected the livers of treated rats and evaluated the therapeutic effect of SWGNS by serological and histological assays. Furthermore, we also analyzed the composition of SWGNS by HPLC. In vitro experiments were conducted to study the protective effect of Crocin, the main component of SWGNS, on BRL-3A cells under peroxide conditions. This is of great significance for understanding the hepatoprotective effect and pharmacological mechanism of SWGNS, which can provide a data basis for its further research and development.

The article "Tibetan Medicine Shi-Wei-Gan-Ning-San Alleviates Carbon Tetrachloride-Induced Chronic Liver Injury by Inhibiting TGF-β1 in Wistar Rats" was published in 2022. Journal: Evid Based Complement Alternat Med.

## 2. Materials and Methods

### 2.1. Ethical

This study was performed in the laboratory of the Hubei Provincial Academy of Preventive Medicine. All procedures involving animals were performed according to Guidelines for the Care and Use of Laboratory Animals and were approved by the Institutional Animal Care and Use Committee (IACUC) (Permit No. 2015021). Animals were allowed to acclimate at least for one week before being subjected to experimental procedures. Wistar rats were purchased from Hubei Experimental Animal Research Center (license number: SCXK (Hubei) 2015–0018). Animals were allowed to acclimate at least for one week before being subjected to experimental procedures. The animals were housed in an IVC cage with 40 air exchanges/h. All the cages were placed in a controlled room with temperature (20–25°C), humidity (40%–70%), and light (a 12 h light/dark cycle).

### 2.2. Reagents

CCl_4_ was purchased from Aladdin (C131583, Shanghai, China). Peanut oil was obtained from Beijing Bailinway Technology Co., Ltd. (C805618, Beijing, China). Enzyme-linked immunosorbent assay (ELISA) kits for TGF-*β*1 (EK0514), rabbit anti-*α*-SMA polyclonal antibody (BM3902), and SABC (rabbit IgG)-AP Kit (SK1052) were purchased from Boster Biological Technology Co., Ltd. (Wuhan, China). HA, LN, and collagen type IV (CIV) radiation immunoassay kit was obtained from Beijing North Biotechnology Research Institute Co., Ltd. (Beijing, China). Assay kits for alanine aminotransferase (ALT, L202360), aspartate aminotransferase (AST, L206360), total protein (TP, L145360), albumin (ALB, L103360), total bilirubin (TBIL, L310220), and gamma-glutamyltransferase (*γ*-GGT, L233300) were provided by Shanghai Huifeng Medical Technology Co., Ltd. (Shanghai, China). CCK-8 kit (G4103) was from Wuhan Servicebio. Malondialdehyde (MDA, A003-1-2) and superoxide dismutase (SOD, A001-3-2) kits were purchased from Nanjing Jiancheng Institute. Bifendate pill was purchased from Beijing Union Pharm. The test article SWGNS formula (Table 1) was provided by the Tibetan Hospital of Tibet Autonomous Region. SWGNS powder and positive control bifendate were, respectively, dissolved to the desired concentration with 0.5% sodium carboxymethyl cellulose (SCC) solution. The formulations were stored in black plastic bottles at 4°C and prepared weekly.

The article "Tibetan Medicine Shi-Wei-Gan-Ning-San Alleviates Carbon Tetrachloride-Induced Chronic Liver Injury by Inhibiting TGF-β1 in Wistar Rats" was published in 2022. Journal: Evid Based Complement Alternat Med.

### 2.3. Animals

78 male Wistar rats aged 4-5 weeks were used for chronic liver injury experiments. Models of CCl_4_-induced chronic liver injury refer to previous studies [12,13]. The animals were randomly divided into 6 groups of 13 rats each. Group 1 served as a blank control and was administrated with vehicle (0.5% SCC) only. Group 2 served as a CCl_4_ model group and was also gavaged with 0.5% SCC. Group 3 served as a positive control and was gavaged with bifendate (100 mg/kg/day). Groups 4, 5, and 6 were treated with SWGNS at three different dose levels (235 mg/kg/day, 705 mg/kg/day, and 1410 mg/kg/day, respectively). SCC, bifendate, and SWGNS were treated by oral gavage once daily for 13 weeks. Meanwhile, animals in groups 2–6 were orally gavaged with 1 mL/kg bodyweight of 50% CCl_4_ peanut oil twice a week for the first 10 weeks and once a week for the last 3 weeks. During week 8, a blood sample was collected from the jugular vein of each animal to monitor biochemistry. After 13 weeks of treatment, the rats were euthanized under phenobarbital, and blood samples and livers were collected for the following tests.

### 2.4. Serum Biochemical Indicators

To detect liver health, serum samples were collected at 3000 RPM at room temperature. Details are as described in previous studies [14,15]. Biomarkers of hepatic injury, alanine aminotransferase (ALT), aspartate aminotransferase (AST), total protein (TP), albumin (ALB), total bilirubin (TBIL), and gamma-glutamyl, transferase (*γ*-GGT) were analyzed by an automatic biochemical analyzer (AU-680, Beckmann, USA). Serum TGF-*β*1 levels were measured using an ELISA kit according to the manufacturer's protocol. The content of HA, LN, and CIV in serum was measured by GC-1200 gamma radioimmunoassay instrument in Wuhan Zhongnan Hospital.

### 2.5. Histopathology

Livers were embedded in paraffin and sectioned to 5 *μ*m thickness. Then, slides were stained with hematoxylin-eosin (H&E). Details are as described in the previous studies [16,17]. Histological changes were observed under a microscope (DM2500, Leica, Germany). Hepatocellular degeneration/steatosis, inflammatory infiltration, necrosis, and fibrosis were evaluated as previously described [18–21]. Lesion scores for each type are as follows: steatosis: 0 (−), no steatosis; 1 (+), steatosis ≤25%; 2 (++), steatosis in 25%–50%; 3 (+++), steatosis ≥50%; inflammatory infiltration: 0 (−), no inflammatory cells infiltration; 1 (+), a small amount of inflammatory cells scattered in the hepatic sinuses, no inflammatory cells in other parts; 2 (++), more inflammatory cells infiltrated in the hepatic lobules and portal areas; 3 (+++), most of the inflammatory cells infiltrated in the hepatic lobules and portal areas; necrosis: 0 (−), no necrotic cells; 1 (+), necrotic cells ≤25%; 2 (++), necrotic cells in 25%–50%; 3 (+++), necrotic cells ≥50%; fibrosis: 0 (−), no fibrosis; 1 (+), slight fibrosis; 2 (++), medium fibrosis, but no pseudolobular formation; 3 (+++), severe fibrosis, visible pseudolobular formation. Total histopathology scores were calculated by summing all scores obtained for each parameter. Liver slides were prepared for immunohistochemical staining with the streptavidin-biotinidase complex (SABC) method according to the manufacturer's protocol.

The article "Tibetan Medicine Shi-Wei-Gan-Ning-San Alleviates Carbon Tetrachloride-Induced Chronic Liver Injury by Inhibiting TGF-β1 in Wistar Rats" was published in 2022. Journal: Evid Based Complement Alternat Med.

### 2.6. Composition Analysis

The active components of SWGNS were analyzed by high-performance liquid chromatography (HPLC). 1.0 g of SWGNS powder was dissolved in 50 mL of 50% methanol in an ultrasonic waterbath for 20 min, and the filtrate was collected for analysis. All the samples were analyzed on octadecyl chemically bonded phase silica gel using methanol as mobile phase A and 0.1% trifluoroacetic acid in water as mobile phase B. The separation was achieved using the following gradient program: 0–25 min, 55% B; 25–45 min, 55–30% B; 45–50 min, 30–55% B; 50–60 min, 55% B. The flow rate was set at 1.0 mL/min, and the injection volume was 10 *μ*L. The detection wavelength was kept at 440 nm. Standard controls Crocin I and Crocin II were purchased from China National Institute for Food and Drug Control. Prepare standard control stock solutions containing 30 *μ*g/mL of Crocin I and 12 *μ*g/mL of Crocin II in 50% methanol. The HPLC method for quantitative and qualitative analyses was according to previous literature (Chinese Pharmacopoeia).

### 2.7. Cell Culture

Rat hepatocyte cell line BRL-3A (CL0376, Fenghui, Changsha, China) was cultured in H-DMEM (C11995500BT, Gibco, USA)+10% FBS (B21001, QuaCell, Zhongshan, China)+1% penicillin-streptomycin (G4003, Servicebio, Wuhan, China) medium at 37°C with 5% CO_2_. The experiments were divided into four groups: control group, H_2_O_2_ group (200 nmol/L), low-dose (1 *μ*g/mL), medium-dose (2 *μ*g/mL), and high-dose (5 *μ*g/mL) treatment groups of Crocin. The control group was cultured normally with DMEM; the H_2_O_2_ group was treated with H_2_O_2_ for 1 hour and then replaced with DMEM for 24 hours. The Crocin-treated groups were changed to DMEM medium containing Crocin after H_2_O_2_pretreatment. Drug concentrations were used as per previous studies [22,23]. Cell viability was detected with a 96-well plate and CCK-8 kit. ALT, AST, MDA, and SOD were measured with ELISA kits. An instruction manual was followed for the detection method.

### 2.8. Statistics

All measurement data are expressed as mean ± SEM. Statistics were performed using SPSS 17 (SPSS Science Inc., Chicago, Illinois, USA). Analysis of variance (ANOVA) was used to compare differences in multiple groups with a post-hoc LSD test. Histopathological scores were analyzed with Kruskal–Wallis and Mann–Whitney tests. Student's unpaired *t*-test was used to compare differences between the two groups. *P* < 0.05 was considered significant. More significant differences are described in the legends.

The article "Tibetan Medicine Shi-Wei-Gan-Ning-San Alleviates Carbon Tetrachloride-Induced Chronic Liver Injury by Inhibiting TGF-β1 in Wistar Rats" was published in 2022. Journal: Evid Based Complement Alternat Med.

## 3. Results

### 3.1. SWGNS Restored CCl_4_-Induced Weight Loss

Bodyweight is a sensitive indicator of animal growth. As shown in Figure 1, compared with the control group, the CCl_4_-treated rats showed a significant decrease in bodyweight right after day 12 of dosing (*P* < 0.01 or *P* < 0.05). However, SWGNS significantly reduced bodyweight loss in rats. In particular, in the SWGNS-fed group at a dose of 705 mg/kg, bodyweight almost returned to normal levels from day 74. The positive control bifendate had little effect on bodyweight improvement.

### 3.2. SWGNS Ameliorated CCl_4_-Induced Decline in Liver Function

To understand whether SWGNS can improve CCl_4_-induced liver injury, the biomarkers of liver injury ALT, AST, TP, ALB, TBIL, and *γ*-GGT were measured in serum. As shown in Figure 2, compared with the control group, the serum levels of ALT, AST, TBIL, and *γ*-GGT of CCl_4_-treated rats were significantly increased, and the levels of TP and ALB were significantly decreased (*P* < 0.01). However, compared with the CCl_4_-treated model group, TBIL and *γ*-GGT levels were significantly decreased in SWGNS-treated groups in a dose-dependent manner (*P* < 0.05 or *P* < 0.01). In addition, ALB levels at weeks 8 and 13 and TP levels at week 13 were significantly recovered (*P* < 0.05 or *P* < 0.01). Serum biochemical results indicated that SWGNS had significant hepatoprotective ability against CCl_4_-induced liver injury.

### 3.3. SWGNS Alleviated CCl_4_-Induced Liver Pathological Changes

To understand the role of SWGNS in alleviating CCl_4_-induced hepatic pathological changes, hepatic pathological changes were assessed. As shown in Figure 3, the histological evaluation results showed that SWGNS reduced CCl_4_-induced liver fibrosis. Histopathological examination of CCl_4_-treated rats showed that the histological changes of chronic liver injury were mainly characterized by severe hepatic steatosis and fibrosis, as well as mild inflammatory infiltration and necrosis. In contrast, CCl_4_-induced liver injury was significantly improved in all rats pretreated with SWGNS. These histopathological data were consistent with serum biochemical results. It suggests that SWGNS can alleviate CCl_4_-induced liver fibrosis.

The article "Tibetan Medicine Shi-Wei-Gan-Ning-San Alleviates Carbon Tetrachloride-Induced Chronic Liver Injury by Inhibiting TGF-β1 in Wistar Rats" was published in 2022. Journal: Evid Based Complement Alternat Med.

### 3.4. SWGNS Ameliorated CCl_4_-Induced Liver Injury by Inhibiting TGF-*β*1 Expression

To understand whether the liver fibrosis alleviated by SWGNS is related to the TGF-*β*1 pathway, the expression of TGF-*β*1, hyaluronic acid, laminin, and collagen IV in serum was measured. As shown in Figures 4(a) and 4(b), TGF-*β*1 and hyaluronic acid were significantly elevated in the CCl_4_-induced chronic liver injury model; and the SWGNS decreased the level of TGF-*β*1 and hyaluronic acid. However, as for laminin and collagen IV, there were no significant differences between the groups (Figures 4(c) and 4(d)). Furthermore, the expression of *α*-SMA was also examined by immunohistochemistry. As shown in Figure 4(e), the expression of *α*-SMA was increased in the CCl_4_ model group, and the increased expression level was inhibited by SWGNS.

### 3.5. Analysis of SWGNS Composition

SWGNS mainly consists of 12 herbs and minerals. We successfully characterized them, especially Crocin I and Crocin II, by HPLC. HPLC results showed that the linear ranges of Crocin I and Crocin II were 3.33–66.67 *μ*g/mL (0.9998) and 1.21–24.24 *μ*g/mL (0.9998), respectively (Figure 5(a)). The mean recovery of Crocin I was 96.50% with an RSD of 1.62%, and the mean recovery of Crocin II was 90.41% with an RSD of 1.85% (Figure 5(b)). It shows that the established HPLC method has high sensitivity, accuracy, and good repeatability and is suitable for the determination of SWGNS phytochemical characteristics. The contents of Crocin I and Crocin II in the samples were 0.23% and 0.07%, respectively.

### 3.6. Crocin Attenuated H_2_O_2_-Induced BRL-3A Cell Injury

Previous studies have reported that Crocin have anti-inflammatory and antioxidant effects [23,24]. Inflammation is a major source of oxidative stress. We investigated the antioxidant protective effect of Crocin through in vitro experiments. The results showed that Crocin increased the cell viability of BRL-3A after H_2_O_2_ pretreatment in a concentration-dependent manner. Further studies showed that Crocin reduced the expression of ALT, AST, MDA, and SOD. It is suggested that Crocin may protect liver cells through their antioxidant effect (Figure 6).

## 4. Discussion

As a traditional Tibetan medicine, SWGNS has been mainly used to treat liver diseases for many years. Many Tibetan medicines have shown obvious advantages in the treatment of liver diseases; and the commonly used natural products include *Carthamus tinctorius, Crocus sativus, Meconopsis integrifolia, Brag-zhun, Herpetospermum pedunculosum*, and *Phyllanthus emblica* [8], which are all included in our SWGNS formula. This study found that SWGNS can alleviate the process of CCl_4_-induced chronic liver injury, such as preventing weight loss, reducing liver injury biomarkers, and improving liver tissue lesions. Additionally, SWGNS may prevent liver pathology by reducing TGF-*β*1 secretion, inflammation, and oxidative stress, which indicates that it has a hepatoprotective effect.

The article "Tibetan Medicine Shi-Wei-Gan-Ning-San Alleviates Carbon Tetrachloride-Induced Chronic Liver Injury by Inhibiting TGF-β1 in Wistar Rats" was published in 2022. Journal: Evid Based Complement Alternat Med.

The dosage of herbal medicine is the key to the treatment. The clinical dose of SWGNS is 1.5 g, 2 times a day, so the dosage is 3.0 g/day. In this study, the calculated dose, such as low, medium, and high, was 1, 3, and 6 times the clinically equivalent dose, respectively. According to the conversion formula of body surface area and bodyweight [lgS (surface) = 0.8762 + 0.698 lgW (weight)], the three-dose levels were calculated as 235, 705, and 1410 mg/kg in rats, respectively. All of these SWGNS doses demonstrated their protective effect in the treatment of chronic liver injury models, especially in liver fibrosis. Furthermore, the therapeutic effect was dose-dependent.

Serum ALT and AST have been the commonly used biomarkers of liver injury, and their release from hepatocytes into the circulation is proportional to the degree of hepatocyte injury [25]. An interesting finding in this study is that the serum ALT and AST levels were significantly increased in the CCl_4_ model group at the early stage (week 8), but no significant changes were observed at the end stage (week 13). Asymptomatic liver fibrosis with normal ALT and AST has been reported clinically [26]. Regardless, prophylactic treatment of SWGNS restored AST and ALT levels in animal models. In addition, SWGNS improved other serum liver function biomarkers, including *γ*-GGT, TBIL, and ALB, which further demonstrated its hepatoprotective activity.

Histopathological evaluation is an important method for the treatment and prognosis of chronic liver disease [27, 28]. Our findings suggest that CCl_4_-induced chronic liver injury is characterized by liver fibrosis, whereas SWGNS reduces the incidence and extent of steatosis and fibrosis. In contrast, although bifendate significantly reduced ALT levels, it did not attenuate histopathological changes. This suggests that SWGNS may have more therapeutic potential than other traditional liver injury drugs.

Fibrosis is the final common histological change in chronic liver disease, characterized by excessive deposition and reorganization of the ECM [29]. Biomarkers of ECM synthesis include HA, LN, and CIV [30,31]. Furthermore, upon HSC activation, they lose vitamin A-containing lipid droplets and transdifferentiate into myofibroblasts that express high *α*-SMA [32]. Thus, these parameters reflect the stage of liver fibrosis. In our model, the levels of HA and *α*-SMA increased significantly in the CCl_4_ model group, whereas the levels of LN and CIV did not change. It has been reported that HA is a sensitive biomarker of early liver fibrosis, and LN and CIV are biomarkers of a later stage [33], which explains our results. We observed that SWGNS significantly decreased HA and *α*-SMA in a dose-dependent manner, implying that SWGNS could inhibit ECM synthesis. TGF-*β* is a central mediator of the liver fibrosis process, activating transdifferentiation from HSCs to myofibroblasts and producing ECM. Previous animal studies demonstrated that hepatic TGF-*β* overexpression increased fibrosis, whereas TGF-*β* neutralization abolished this process [34–36]. Therefore, anti-TGF-*β* strategies have been developed to treat chronic liver diseases [37]. Here, we further demonstrated that SWGNS may prevent liver fibrosis by inhibiting TGF-*β*1.

The article "Tibetan Medicine Shi-Wei-Gan-Ning-San Alleviates Carbon Tetrachloride-Induced Chronic Liver Injury by Inhibiting TGF-β1 in Wistar Rats" was published in 2022. Journal: Evid Based Complement Alternat Med.

Previous studies have demonstrated that excessive inflammation and ROS are important causes of liver injury, and inhibiting inflammation and ROS can effectively alleviate liver injury [38–42]. Especially in the CCl_4_-induced liver injury model, several studies indicate that natural products can alleviate tissue injury by modulating immune responses and oxidative stress [43–46]. TGF-*β*1 is well known for regulating inflammation and oxidative stress [47,48]. In other words, TGF-*β*1 can be associated with the process of liver injury by mediating inflammation and oxidative stress, for example, downregulation of miR-10a can suppress sepsis-induced liver injury by downregulating the TGF-*β*1 pathway, as well as inflammation and oxidative stress [49]. Silymarin can alleviate CCl_4_-induced liver injury by inhibiting oxidative stress, inflammation, and TGF-*β*1 [50]. The study also indicates that oxidative stress is a key factor driving inflammation and TGF-*β*1. Our view/results are parallel to the previous literature. Since there are more studies on inflammation and oxidative stress, we paid more attention to the changes in TGF-*β*1. We hypothesized that SWGNS significantly downregulated the expression of TGB-*β*1 in vivo and that Crocin significantly reduced oxidative stress in vitro. Therefore, we believe that SWGNS protects the liver by reducing TGF-*β*, inflammation, and oxidative stress.

This study has some limitations. First, toxicity testing has not been performed. The composition of herbal medicines is complex, and in addition to the effective components, there is the possibility of toxic components. Further testing of the effects of SWGNS on other organs is required. Second, there is a lack of dose testing: we tested the effect of SWGNS at three different doses and found that its liver-protective effect was dose-dependent. However, higher doses may have unpredictable side effects. Therefore, verification is required. Furthermore, more active ingredients for liver protection need to be identified. In the future, we are planning to isolate more active ingredients to further characterize their effects and toxicity because this will be more important for mass production and promotion. In addition, numerous studies have shown that herbal medicines generally have anti-inflammatory and antioxidant effects, which is one of the key mechanisms of treatment. SWGNS also has anti-inflammatory and antioxidant effects, but lack of in-depth mechanism research. This is also the focus of future research.

The article "Tibetan Medicine Shi-Wei-Gan-Ning-San Alleviates Carbon Tetrachloride-Induced Chronic Liver Injury by Inhibiting TGF-β1 in Wistar Rats" was published in 2022. Journal: Evid Based Complement Alternat Med.

## 5. Conclusions

In conclusion, this study demonstrates that SWGNS reduces CCl_4_-induced chronic liver injury by inhibiting TGF-*β*1 expression for the first time. Also, it shows that SWGNS is a promising drug for the treatment of liver fibrosis, which is worthy of further research, development, and promotion.

## Figures and Tables

**Figure 1:** SWGNS formula recovered the bodyweight of the CCl_4_-treated rats. ^#^*P* < 0.05. ^##^*P* < 0.01. The CCl_4_-induced model group versus the normal control group.^*∗*^*P* < 0.05. ^*∗∗*^*P* < 0.01. SWGNS at 705 mg/kg treated rats versus the CCl_4_-induced model group (*n* = 10–13 each group).

**Figure 2:** SWGNS improved enzymatic activity of ALT, AST, and *γ*-GGT and the levels of TP, ALB, and TBIL in the CCl_4_-induced hepatic fibrosis. ^#^*P* < 0.05 and ^##^*P* < 0.01 versus the normal control group; ^*∗*^*P* < 0.05 and ^*∗∗*^*P* < 0.01 versus the CCl_4_-induced model group (*n* = 10–13 each group).

**Figure 3:** SWGNS alleviated CCl_4_-induced liver pathological changes. (a) Representative photos of H&E staining. 200X magnification.(a) normal control; (b) CCl_4_ model control; (c) CCl_4_+ bifendate at 200 mg/kg; (d) CCl_4_+ SWGNS at 235 mg/kg; (e) CCl_4_+ SWGNS at 705 mg/kg; (f) CCl_4_+ SWGNS at 1410 mg/kg. (b) Histopathology scores of each group. ^##^*P* < 0.01 versus the normal control group, ^*∗*^*P* < 0.05. ^*∗∗*^*P* < 0.01 versus the CCl_4_ model group (*n* = 13 each group).

**Figure 4:** SWGNS protects against CCl_4_-induced liver injury by mediating TGF-*β*1. (a) Serum TGF-*β*1 concentration; (b) serum HA concentration; (c) serum LN concentration; (d) serum CIV concentration. ^*∗*^*P* < 0.05 and ^*∗∗*^*P* < 0.01, compared to the CCl4 model group. *n* = 10–13. (e) Representative photos of *α*-SMA in the liver section. (a) Blank control; (b) CCl4 model group; (c) CCl4+ bifendate at 200 mg/kg; (d) CCl4+ SWGNS at 235 mg/kg; (e) CCl4 + SWGNS at 705 mg/kg; (f) CCl_4_+ SWGNS at 1410 mg/kg. 100X magnification.

The article "Tibetan Medicine Shi-Wei-Gan-Ning-San Alleviates Carbon Tetrachloride-Induced Chronic Liver Injury by Inhibiting TGF-β1 in Wistar Rats" was published in 2022. Journal: Evid Based Complement Alternat Med.

**Figure 5:** The HPLC chromatogram of standard Crocin I and II sample (a) and SWGNS sample (b). 1, Crocin I; 2, Crocin II.

**Figure 6:** The role of Crocin in protecting BRL-3A cells from a peroxidative environment. (a) Cell viability. (b) ALT. (c) AST. (d) MDA.(e) Total SOD. ^#^*P* < 0.05, compared to the control group.^*∗*^*P* < 0.05, compared to the H_2_O_2_ group. *n* = 5.

**Table 1:** The composition of Tibetan medicine SWGNS formula.

English name	Chinese name	Source	Amount (%)
*Carthamus tinctorius*	Honghua	Dry flowers of *Carthamus tinctorius* L	70 g (13%)
*Crocus sativus*	Fanhonghua	The dry stigma of *Crocus sativus* L	15 g (2.8%)
*Herpetospermum pedunculosum*	Bolengguazi	Dried seeds of *Herpetospermum pedunculosum* (Ser.) Baill	50 g (9.3%)
*Meconopsis integrifolia*	Lvronghao	The dried whole grass of *Meconopsis integrifolia* (Maxim.) Franch, *Meconopsis quintuplinervia* Regel, and *Meconopsis lancifolia* (Franch.) Franch	70 g (13%)
*Dracocephalum tanguticum*	Ganqingqinglan	The dry aboveground part of *Dracocephalum tanguticum* Maxim	70 g (13%)
*Saxifraga stolonifera*	Lianzuohuercao	*Saxifraga pasumensis*, a plant of the genus snail Marq.et Dry whole grass of *Saxifraga confertifolia* Engl. and *Saxifraga candelabrum* Franch.	50 g (9.3%)
*Corydalis impatiens*	Zijin	The dried whole plant of *Corydalis hendersonii* Hemsl. (*c. nepaiesis* Kitamura) and *c. mucionifera* Maxim.	50 g (9.3%)
Bear gallbladder	Xiongdanfen	The dried product of *Selenarctos thibetanus* Cuvier, a bear in the family Ursidae, which is drained bile by gallbladder operation	0.5 g (0.093%)
Calculus Bovis	Niuhuang	Gallstones in the gallbladder of *Bos taurus domesticus* Gmelin	1.0 g (0.186%)
Brag-zhun	Zhaxungao	The cream is made from the dry feces of *Trogopterus xanthipes* Milne Edwards	50 g (9.3%)
Calciosinti	Shihuihua	Carbonate minerals, mainly containing calcium carbonate (CaCO_3_)	50 g (9.3%)
Turquoisis	Songshi	A mineral formed by the precipitation of copper-bearing aqueous solution with alumina-bearing minerals and phosphorus-bearing minerals in fractures under supergene conditions. The main water-bearing phosphate containing copper and aluminum is CuAl_6_ (PO_4_)_4_ (OH)_8_·4H_2_O.	60 g (11%)

## Data Availability

The data used to support the findings of this study are available from the corresponding author upon request.

## References

[1] Wang F. S., Fan J. G., Zhang Z., Gao B., Wang H. Y. (2014). The global burden of liver disease: the major impact of China. *Hepatology*.

[2] Ain Q. T. (2021). Hepatotoxicity induced by intravenous administration of PEGylated nano-graphene oxide in albino mice. *Materials Express*.

The article "Tibetan Medicine Shi-Wei-Gan-Ning-San Alleviates Carbon Tetrachloride-Induced Chronic Liver Injury by Inhibiting TGF-β1 in Wistar Rats" was published in 2022. Journal: Evid Based Complement Alternat Med.

[3] Yu X., Pan J., Shen N. (2021). Development of saikosaponin D liposome nanocarrier with increased hepatoprotective effect against alcoholic hepatitis mice. *Journal of Biomedical Nanotechnology*.

[4] Choi D. J., Kim S. C., Park G. E. (2020). Protective effect of a mixture of Astragalus membranaceus and lithospermum erythrorhizon extract against hepatic steatosis in high fat diet-induced nonalcoholic fatty liver disease mice. *Evidence-Based Complementary and Alternative Medicine*.

[5] Romanelli R. G., Stasi C. (2016). Recent advancements in diagnosis and therapy of liver cirrhosis. *Current Drug Targets*.

[6] Barcena-Varela M., Colyn L., Fernandez-Barrena M. G. (2019). Epigenetic mechanisms in hepatic stellate cell activation during liver fibrosis and carcinogenesis. *International Journal of Molecular Sciences*.

[7] Chen T., Zhu C., Wang X., Pan Y., Huang B. (2021). Asiatic acid encapsulated exosomes of hepatocellular carcinoma inhibit epithelial-mesenchymal transition through transforming growth factor beta/smad signaling pathway. *Journal of Biomedical Nanotechnology*.

[8] Li Q., Li H. J., Xu T. (2018). Natural medicines used in the traditional Tibetan medical system for the treatment of liver diseases. *Frontiers in Pharmacology*.

[9] Feng X., Li M. H., Xia J. (2018). Tibetan medical formula shi-wei-Gan-Ning-Pill protects against carbon tetrachloride-induced liver fibrosis - an NMR-based metabolic profiling. *Frontiers in Pharmacology*.

[10] Wang Q. (2018). Effect of Tibetan medicine Shiwei Ganning powder on transaminase elevation induced by alcoholic liver injury. *Journal of Medicine & Pharmacy of Chinese Minorities*.

[11] Kan Z. (2014). Cases study of “shiweiganning powder” in the treatment of fatty liver disease. *China Tibetology*.

[12] Dai N., Zou Y., Zhu L., Wang H. F., Dai M. G. (2014). Antioxidant properties of proanthocyanidins attenuate carbon tetrachloride (CCl4)-induced steatosis and liver injury in rats via CYP2E1 regulation. *Journal of Medicinal Food*.

[13] Cho B. O., Ryu H. W., So Y. (2013). Hepatoprotective effect of 2, 3-dehydrosilybin on carbon tetrachloride-induced liver injury in rats. *Food Chemistry*.

[14] Gigliotti J. C., Tin A., Pourafshar S. (2020). GSTM1 deletion exaggerates kidney injury in experimental mouse models and confers the protective effect of cruciferous vegetables in mice and humans. *Journal of the American Society of Nephrology*.

[15] Jin T., Wang L., Li D., Yang T., Zhou Y. (2020). Testosterone aggravates cerebral vascular injury by reducing plasma HDL levels. *Open Life Sciences*.

[16] Wang M., Yao S., He D. (2020). Type 2 diabetic mellitus inhibits skin renewal through inhibiting WNT-dependent Lgr5+ hair follicle stem cell activation in C57BL/6 mice. *Journal of Diabetes Research*.

The article "Tibetan Medicine Shi-Wei-Gan-Ning-San Alleviates Carbon Tetrachloride-Induced Chronic Liver Injury by Inhibiting TGF-β1 in Wistar Rats" was published in 2022. Journal: Evid Based Complement Alternat Med.

[17] Meng F., Qiu J., Chen H. (2021). Dietary supplementation with N-3 polyunsaturated fatty acid-enriched fish oil promotes wound healing after ultraviolet B induced sunburn in mice. *Food Sciences and Nutrition*.

[18] Kirac E., Ozcan F., Tuzcu H., Elpek G. O., Aslan M. (2015). Analysis of polyunsaturated fatty acids and the omega-6 inflammatory pathway in hepatic ischemia/re-perfusion injury. *Molecular Medicine Reports*.

[19] Yang G., Istas G., Hoges S. (2018). Angiotensin-(1-7)-induced Mas receptor activation attenuates atherosclerosis through a nitric oxide-dependent mechanism in apolipoproteinE-KO mice. *Pfluegers Archiv European Journal of Physiology*.

[20] Stegbauer J., Thatcher S. E., Yang G. (2019). Mas receptor deficiency augments angiotensin II-induced atherosclerosis and aortic aneurysm ruptures in hypercholesterolemic male mice. *Journal of Vascular Surgery*.

[21] Hammer A., Yang G., Friedrich J. (2016). Role of the receptor Mas in macrophage-mediated inflammation in vivo. *Proceedings of the National Academy of Sciences*.

[22] Kopalli S. R., Cha K. M., Cho J. Y., Kim S. K., Koppula S. (2022). Cordycepin mitigates spermatogenic and redox related expression in H(2)O(2)-exposed Leydig cells and regulates testicular oxidative apoptotic signalling in aged rats. *Pharmaceutical Biology*.

[23] Zhao T., Lu H., Li M., Yan Q., Gu J., Liu L. (2022). Neuroprotective mechanism of crocin via PI3K/Akt/mTOR signaling pathway after cerebral infarction: an in vitro study. *American Journal of Translational Research*.

[24] Zhu K., Yang C., Dai H. (2019). Crocin inhibits titanium particle-induced inflammation and promotes osteogenesis by regulating macrophage polarization. *International Immunopharmacology*.

[25] McGill M. R. (2016). The past and present of serum aminotransferases and the future of liver injury biomarkers. *EXCLI J*.

[26] Beaton M., Adams P. C. (2008). Assessment of silent liver fibrosis in hemochromatosis C282Y homozygotes with normal transaminase levels. *Clinical Gastroenterology and Hepatology*.

[27] Straub B. K., Schirmacher P. (2010). Pathology and biopsy assessment of non-alcoholic fatty liver disease. *Digestive Diseases*.

[28] Bedossa P. (2017). Pathology of non-alcoholic fatty liver disease. *Liver International*.

[29] Parola M., Pinzani M. (2019). Liver fibrosis: pathophysiology, pathogenetic targets and clinical issues. *Molecular Aspects of Medicine*.

[30] Gudowska M., Cylwik B., Chrostek L. (2017). The role of serum hyaluronic acid determination in the diagnosis of liver fibrosis. *Acta Biochimica Polonica*.

The article "Tibetan Medicine Shi-Wei-Gan-Ning-San Alleviates Carbon Tetrachloride-Induced Chronic Liver Injury by Inhibiting TGF-β1 in Wistar Rats" was published in 2022. Journal: Evid Based Complement Alternat Med.

[31] Gulubova M. V., Vlaykova T. I. (2006). Significance of tenascin-C, fibronectin, laminin, collagen IV, alpha5beta1 and alpha9beta1 integrins and fibrotic capsule formation around liver metastases originating from cancers of the digestive tract. *Neoplasma*.

[32] Kinnman N., Goria O., Wendum D. (2001). Hepatic stellate cell proliferation is an early platelet-derived growth factor-mediated cellular event in rat cholestatic liver injury. *Laboratory Investigation*.

[33] Stickel F., Poeschl G., Schuppan D. (2003). Serum hyaluronate correlates with histological progression in alcoholic liver disease. *European Journal of Gastroenterology and Hepatology*.

[34] Ling H., Roux E., Hempel D. (2013). Transforming growth factor beta neutralization ameliorates pre-existing hepatic fibrosis and reduces cholangiocarcinoma in thioacetamide-treated rats. *PLoS One*.

[35] Li H., Li Q., Zhang X., Zheng X., Zhang Q., Hao Z. (2018). Thymosin *β*4 suppresses CCl_4_-induced murine hepatic fibrosis by down-regulating transforming growth factor *β* receptor-II. *The Journal of Gene Medicine*.

[36] Du S. S., Qiang M., Zeng Z. C. (2010). Radiation-induced liver fibrosis is mitigated by gene therapy inhibiting transforming growth factor-beta signaling in the rat. *International Journal of Radiation Oncology, Biology, Physics*.

[37] Breitkopf K., Haas S., Wiercinska E., Singer M. V., Dooley S. (2005). Anti-TGF-beta strategies for the treatment of chronic liver disease. *Alcoholism: Clinical and Experimental Research*.

[38] Sadek K. M., Lebda M. A., Abouzed T. K., Nasr S. M., El-Sayed Y. (2018). The molecular and biochemical insight view of lycopene in ameliorating tramadol-induced liver toxicity in a rat model: implication of oxidative stress, apoptosis, and MAPK signaling pathways. *Environmental Science and Pollution Research*.

[39] Sadek K., Abouzed T., Nasr S., Shoukry M. (2020). Licochalcone B ameliorates liver cancer via targeting of apoptotic genes, DNA repair systems, and cell cycle control. *Iranian Journal of Pharmaceutical Research*.

[40] Liu Z. G., Qian X., Wang Z. M. (2021). Effects of persimmon tannin-aloe vera composite on cytotoxic activities, and radioprotection against X-rays irradiated in human hepatoma and hepatic cells. *Journal of Biomedical Nanotechnology*.

[41] Munakarmi S., Chand L., Shin H. B., Jang K. Y., Jeong Y. J. (2020). Indole-3-Carbinol derivative DIM mitigates carbon tetrachloride-induced acute liver injury in mice by inhibiting inflammatory response, apoptosis and regulating oxidative stress. *International Journal of Molecular Sciences*.

[42] Zhang Y., Wang C., Bai Z., Li P. (2021). Umbilical cord mesenchymal stem cell exosomes alleviate the progression of kidney failure by modulating inflammatory responses and oxidative stress in an ischemia-reperfusion mice model. *Journal of Biomedical Nanotechnology*.

The article "Tibetan Medicine Shi-Wei-Gan-Ning-San Alleviates Carbon Tetrachloride-Induced Chronic Liver Injury by Inhibiting TGF-β1 in Wistar Rats" was published in 2022. Journal: Evid Based Complement Alternat Med.

[43] Sadek K., Beltagy D., Saleh E., Abouelkhair R. (2016). Camel milk and bee honey regulate profibrotic cytokine gene transcripts in liver cirrhosis induced by carbon tetrachloride. *Canadian Journal of Physiology and Pharmacology*.

[44] Zeweil M. M., Sadek K. M., Elsadek M. F., Mahmoud S. F., Ahmed B. M., Khafaga A. F. (2020). Sidr honey abrogates the oxidative stress and downregulates the hyaluronic acid concentration and gene expression of TGF-*β*1 and COL1a1 in rat model of thioacetamide-induced hepatic fibrosis. *Animal Science Journal*.

[45] Lebda M. A., Sadek K. M., Abouzed T. K., Tohamy H. G., El-Sayed Y. S. (2018). Melatonin mitigates thioacetamide-induced hepatic fibrosis via antioxidant activity and modulation of proinflammatory cytokines and fibrogenic genes. *Life Sciences*.

[46] Sadek K. M., Saleh E. A., Nasr S. M. (2018). Molecular hepatoprotective effects of lipoic acid against carbon tetrachloride-induced liver fibrosis in rats: hepatoprotection at molecular level. *Human & Experimental Toxicology*.

[47] Wahl S. M. (1992). Transforming growth factor beta (TGF-beta) in inflammation: a cause and a cure. *Journal of Clinical Immunology*.

[48] Chen H. Y., Chou H. C., Ho Y. J. (2021). Characterization of TGF-*β* by induced oxidative stress in human trabecular meshwork cells. *Antioxidants*.

[49] Zhou Y. X., Han W. W., Song D. D. (2020). Effect of miR-10a on sepsis-induced liver injury in rats through TGF-*β*1/Smad signaling pathway. *European Review for Medical and Pharmacological Sciences*.

[50] Al-Rasheed N., Faddah L., Al-Rasheed N. (2016). Protective effects of silymarin, alone or in combination with chlorogenic acid and/or melatonin, against carbon tetrachloride-induced hepatotoxicity. *Pharmacognosy Magazine*.

